The article "Automatic Building Extraction on Satellite Images Using Unet and ResNet50" was published in 2022. Journal: Comput Intell Neurosci.

# Automatic Building Extraction on Satellite Images Using Unet and ResNet50

**DOI:** 10.1155/2022/5008854

**Published:** 2022-02-18

**Authors:** Waleed Alsabhan, Turky Alotaiby

**Affiliations:** King Abdulaziz City for Science and Technology, National Center for Data Analytics and Artificial Intelligence, P.O. Box 6086, Riyadh 11442, Saudi Arabia

## Abstract

Recently, settlement planning and replanning process are becoming the main problem in rapidly growing cities. Unplanned urban settlements are quite common, especially in low-income countries. Building extraction on satellite images poses another problem. The main reason for the problem is that manual building extraction is very difficult and takes a lot of time. Artificial intelligence technology, which has increased significantly today, has the potential to provide building extraction on high-resolution satellite images. This study proposes the differentiation of buildings by image segmentation on high-resolution satellite images with U-net architecture. The open-source Massachusetts building dataset was used as the dataset. The Massachusetts building dataset includes residential buildings of the city of Boston. It was aimed to remove buildings in the high-density city of Boston. In the U-net architecture, image segmentation is performed with different encoders and the results are compared. In line with the work done, 82.2% IoU accuracy was achieved in building segmentation. A high result was obtained with an F1 score of 0.9. A successful image segmentation was achieved with 90% accuracy. This study demonstrated the potential of automatic building extraction with the help of artificial intelligence in high-density residential areas. It has been determined that building mapping can be achieved with high-resolution antenna images with high accuracy achieved.

## 1. Introduction

Less-developed countries, especially in Asia and Africa, often witness new unplanned settlements like slums, urban villages, and shantytowns as the urban sprawls continue to cater to the increasing population [1]. The statistics for this problem can be known by the mapping of the settlements for nearly 564 million rural population in China [2]. There is a rapidly increasing demand for housing facilities for the low-income population. This demand has led to the settlement of many unplanned areas, which are highly packed with small buildings [3]. While these unplanned settlements do provide housing for low-income personals, they have become to the root causes of unequal and unsatisfactory living conditions and standards. Moreover, the public safety sector has been majorly compromised [4]. These situations require efficient management, reconstruction, and big leap improvement of unplanned habitats. To devise a strategic policy, it is important to understand every component that prepares the area and every construction that characterizes the slum [5]. Urban villages are the most common outcomes of the discussed urban sprawling worldwide and require immediate attention. Traditional methods of cartography of unplanned construction in urban settlements require field visits, extensive measurement of constructions of interest, and manual digitalization of data. This field survey requires high manpower and expenses because of the increasing complexity and number of urban villages. Remote sensing provides a less easy, less costly, and more accurate alternative to field surveys that allow larger coverage. Consequently, it is a perfect method to update databases if employed wisely. Manually classifying objects taken from low altitudes and via Unmanned Aerial Vehicle imaging technology is also severely extensive despite some advantages over field surveys. The best way forward is to have an automated, intelligent, image-based solution. Some of the latest work on this topic is Refs. [6–9].

This topic covering the mapping of urban settlements based on remote sensing images has a rich history and supporting literature [10]. This problem is being easily dominated by Object-Based Image Analysis (OBIA) of high-resolution optical images [11]. It is common for these solutions to exploit spectral and spatial features for image target identification [12]. Recent works have very confidently relied on Random Forest (RF) for the required building mappings based on machine learning [13]. A lot of many other classification models have been built and tweaked for mapping construction in high-density urban areas, and these pixel- and object-based methods are not useful when we need to extract individual buildings. These methods classify all buildings in one segment or label [14]. When considering complex urban settlements, the features are very hard to define using conventional methods mainly because of the high variance among the buildings [15]. Segmentation is defined as the procedure of grouping pixels into groups based on the similarity in brightness, texture, color, etc. [15]. Common segmentation techniques reach bottlenecks such as scale selection and rule definition when working with high-density images of urban settlements. Completely outlining the boundaries and identifying their shapes are extremely challenging because of high noise and texture elements, which also degrade the performance of the algorithm [16]. As a result, a straightforward and generalized solution is hard to reach and has not been reported in the literature. This means that correct building level segmentation and mapping of unplanned urban settlements are difficult problems for computer vision.

Although there are prominent studies that have segmented slums in remote sensing images based on their differences in physical characteristics from formal settings [17], it is important to go beyond segmenting slums from urban areas and characterize individual buildings for more efficient applications. For example, to know the best strategy for urban reconstruction and its potential benefits, both governmental and private sector people and decision-makers should have adequate information about reconstruction incentives, environmental benefits, and public services [18].

In recent times, deep learning is being applied in an increasing number of domains including computer vision and wireless technologies [19–21], unlike the traditional pixel-based methods [22] like iterative self-organization (ISO) clustering [23], random forest [24], and minimum distance supervision, deep learning methods, and networks can extract multilayer features that can explain abstract and semantic information for potential applications. Consequently, deep learning has become the go-on solution for target detection and classification [25]. Highly efficient models now offer a strong baseline for using deep learning in high-resolution remote sensing (HRRS) applications. The main backbone of deep learning is the neural networks; the most common of them are Convolutional Neural Networks (CNN) [26], Deep Belief Networks (DBN) [27], and Recurrent Neural Networks (RNN) [28]. Different architectures of CNN are already being applied for extracting features in computer vision, Natural Language Processing (NLP), medical imaging, and remote sensing [29]. Remote Sensing Scene Classification (RSSC) returns semantic classes with potential applications in land cover and land-use classification. High-Resolution Remote Sensing (HRRS) is a common example of RSSC and is applied to precision agriculture, urban mapping, natural resource management, and target detection. The last few years have witnessed a lot of endeavors for developing good feature representation and classification models of HSSR images to put them in use in broader areas of implementation. Urban areas have benefited from this progress, and immense improvement has been made in solutions of urban flooding, green space detection [30], hard target identification [31], urban flood [32], and urban pollution (air and water) [33] and has emerged with the occurrence and development of HSRRS imaging [34]. The high-speed development of remote sensing technologies has also helped accelerate the process by allowing the accumulation and generation of benchmark datasets that include: the SAT-4 and SAT-6 airborne datasets [35], the SpaceNet dataset [36], and the UC Merced land-use dataset [37]. These higher resolution images from the HRRS dataset give texture and color information more prominently. Moreover, they contain various scene classes and multiple changes from the traditional images in the domain of remote sensing and are very hard to process if the traditional pixel-based approaches are followed. On the contrary, deep learning networks are capable of classification and object-level recognition of HRRS images and extracting and understanding the contents of these images on the semantic level. These networks can automatically extract features from their deep architectures (for example, CNN and CapsNet) by learning from relevant data [38]. Hence, these magical algorithms have achieved a significant progress in object detection and scene classification. Urban-built area recognition is an important area of computer vision and research top with potential practical applications. While there are traditional techniques already accomplishing the tasks, these techniques do not consider the urban functions [39]. It is more difficult because several built-up areas may have the same construct but different functions. For example, residents and city roads are constructed the same way but have significantly different functions. When considering practical applications, urban planning and emergency planning require functional information and classification. Hence, this category of classification is super important for urban planning, urban ecology, urban emergency, and more.

The remainder of the paper is organized as follows: Introduction and Literature are discussed in Section 1 wherein the problem statement and the current literature work happened on this problem are discussed; Section 2 “Materials and Methods” discusses about the dataset used in this study; then the Methodology section shows the U-net architecture, which is used as implementation steps with all the details; the next section is the Results wherein all the results got after processing are discussed with relevant tables and figure, followed by discussion and conclusion sections giving a brief explanation about the whole process and finally the list of references.

## 2. Materials and Methods

### 2.1. Dataset

The Massachusetts building dataset is published in 2013, and it is among the first publicly available aerial image dataset used for training CNNs [40]. The dataset consists of aerial images of densely populated areas of the city of Boston. It consists of 151 different images. The dataset contains 1500 × 1500 pixels sized images. Each image covers an area of 2.25 km^2^ at a resolution 1 m^2^/pixel. It covers an area of approximately 340 square kilometers. The data are decomposed into 4 images for the validation set, 137 images for the train set, and 10 images for the test set. Building footprints obtained from the OpenStreetMap project were used to label buildings on target maps.

Images of the dataset were restricted to several regions with omission noise levels of less than 5%. Thanks to the OpenStreetMap project, a large amount of high-quality building footprint data were collected. Dataset uses images released by the state of Massachusetts. Images include densely populated areas and include building labels of any size. This dataset is derived from Volodymyr Mnih's original Massachusetts building datasets. Massachusetts Roads and Buildings datasets were introduced in Chapter 6 of his PhD thesis. The total size of dataset is 3 GB. The classes of the dataset are as follows:

1. Background
2. Building

Here is a sample from the dataset with its mask (see Figure 1).

### 2.2. Preprocessing

In this section, preprocessing of the dataset is considered and explained, and preprocessing part is necessary to match our model architectures with the selected dataset.

Each image has masking images to indicate building label (see Figure 2). Masking images are specified as white for buildings and black for the background. Each pixel gets a value for these two different states. These values, which are specified as RGB, are reinforced as [0, 0, 0] for black color and [255, 255, 255] for white color. Here, as a preprocess, masking images are converted as 1 or 0 value instead of RGB value. Thus, the masking image is not used as RGB with 3 layers. Instead, the visuals contain as much depth as the number of classes. In this case, the masking images were converted to HxWx2.

Since the images are very large at 1500 × 1500 × 3 size, it affects the performance badly. In order to ensure a better performance of the model, the images are divided into sections with the size of 256 × 256 × 3 and given in parts. Thus, the performance of the model was increased.

In many artificial intelligence problems, it is necessary to prevent overfitting, increase data diversity, etc. For this purpose, the data augmentation method is applied. In this work, some data augmentation methods were used on the training dataset. Horizontal flip, vertical flip, random rotate 90 degree, added blur, random brightness contrast, and added Gaussian noise data augmentation methods were applied to 50% of the training dataset. Thus, the existing dataset was expanded (see Figure 3), and examples of augmented visuals are given.

### 2.3. Research Methodology

In this part, model architecture is explained in detail.

### 2.4. Model Architecture

In this work, semantic segmentation was developed based on U-net architecture [41] (see Figure 4). UNet, which is a kind of Convolutional Neural Networks (CNN) approach, is first a proposal to make better segmentation on biomedical images. The architecture is effective for the applications that is wanted to obtain the output image size that is similar to the input image size. Therefore, the image is downsampling (encoder) by using Convolution Layers and upsampling (decoder) to obtain the image back with segmentation. The encoder path captures the context of the image producing feature maps. The decoder path is used to enable precise localization using transposed convolutions. As a result, an output of input size and class depth is obtained. Using the U-net architecture, an estimate is made for each pixel of the input picture. This is a very suitable inference for the building extraction task in the work.

U-net has a symmetrical structure. It has two structures, an encoder and a decoder. These structures are connected to each other by skip connections. It can also preserve U-net feature maps in the original image size. The visual of the U-Net architecture made by Ronneberger and her team can be seen in Figure 1. The backbone is the architectural element, which defines how these layers are arranged in the encoder network and they determine how the decoder network should be built. The backbones used are often Vanilla CNNs such as VGG, ResNet, Inception, and EfficientNet, which perform encoding and downsampling by itself. These networks are taken, and their counterparts are built to perform decoding and upsampling to form the final U-Net. This study is based on the U-net model.

Two different models are considered for the exact result (see Figure 5). One of them is to provide feature extraction with a sequential CNN backbone structure, and the other one uses ResNet architecture as a backbone structure. By comparing the training parameters of these two models, the model with the best performance will be presented. ResNet (Residual Network) is a neural network used as a backbone for many computer vision models. Under normal circumstances, training deeper neural networks is quite challenging. There seem to be increased error rates in training deeper neural networks due to the vanishing gradient problem. In theory, training error should decrease when multiple Convolution Neural networks are stacked. However, in practice, it seems that adding more layers to the Convolution Neural Network increases the training error. Optimization or corruption problems occur here.

ResNet solves this problem by resorting to shortcuts. This is a technique called skip connection. Skip connection skips several layers and connects directly to output. In this way, the exploding/vanishing gradient problem is avoided. There are many different ResNet architectures. It is named according to the depth layers (see Figure 6).

There are different variations of the ResNet architecture. It is generally named according to the number of layers. The most widely used ResNet architectures are ResNet34, ResNet50, and ResNet152. With the ImageNet dataset, the model weights trained with millions of datasets can be reached. Using the parameters of the ImageNet dataset as the starting weight for training significantly increases the performance.

## 3. Results

In this section, evaluating metrics for training the model, and obtained results for train, validate, and test processes are considered and explained, respectively. The evaluation metrics are selected with respect to our model architecture.

### 3.1. Evaluation Metrics

#### 3.1.1. Intersection-Over-Union (IoU)

IoU is a metric that is also known as the Jaccard Index, which is widely used in semantic segmentation. IoU is a quite simple evaluation metric that is extremely useful and effective. The overlap area between the IoU predicted segmentation area and the underlying real area is divided by the junction area between the predicted segmentation and the real area. The IoU metric ranged from 0 to 1.0 corresponds to no overlap and 1 corresponds to full overlap. The IoU using dual (two classes) or multiclass segmentation is calculated by taking the average IoU of the image, the IoU of each class, and averaging it as shown in Equation (1). This metric is closely related to the Dice coefficient used as the loss function. Below is the general formula for Intersection-over-Union.

(1) $$\begin{array}{c} \mathrm{IoU}=\frac{\mathrm{target}\cap \mathrm{prediction}}{\mathrm{target}\cap \mathrm{prediction}}. \end{array}$$

Pixels in both the Prediction mask and the actual mask are intersections. All pixels in the prediction and actual mask are unions. The IoU score, calculated separately for each class, is then averaged across all classes to provide a global, average IoU score in our semantic segmentation estimation.

#### 3.1.2. Dice Loss

Dice loss results from the Sørensen–Dice coefficient, a statistic developed in the 1940s to measure similarity between two samples. It was brought to the computer vision community by Milletari et al. It was used for 3D medical image segmentation in 2016. It has also been adapted as a loss function known as Dice Loss. Below is the Dice Loss function:

(2) $$\begin{array}{c} D=\frac{2\sum_{i}^{N}p_{i}g_{i}}{\sum_{i}^{N}p_{i}^{2}+\sum_{i}^{N}g_{i}^{2}}. \end{array}$$

#### 3.1.3. Train, Validate, and Test Results

The whole process includes data loading, preprocessing, and balancing the data followed by data augmentation, and these all steps need high computation power and time. These tasks were accomplished by using Google Colab and the data were downloaded using Google drive. The model training was conducted by working on Graphical Processing Unit (GPU). The main hardware used for this experimentation are GPUs assigned by Google Colab as Tesla P100-PCIEE series 16 GB model and Python 3.9 version is used.

At this stage of the work, three different models were trained, and the accuracy values of these models were compared. One of the models is Unet, which is a fully convolutional neural network for image semantic segmentation. It consists of encoder and decoder parts connected by skip connections. As another model, it is a model that is formed by replacing the encoder part of the Unet model, which consists of fully convolutional neural networks, with the ResNet50 model. As another model, it is a model created by replacing the encoder part of the Unet model, which consists of fully convolutional neural networks, with the ResNet152 model, which is a deeper architecture.

Parameter selection for training is very important for the performance of the model. In this work, the dice loss function, which is very popular in image segmentation problems, was used as a loss function. Dice loss originates from Sørensen–Dice coefficient, which is a statistic developed in the 1940s to gauge the similarity between two samples [43]. Intersection-over-Union function was used to evaluate model performance. The Intersection-over-Union (IoU), also known as the Jaccard Index, is one of the most commonly used metrics in semantic segmentation. The threshold value for the acceptance of accuracy was accepted as 0.5. As the optimizer, Adam optimizer, which has been very popular and effective lately, was chosen.

With the determination of the metrics, first of all, training was carried out on the Unet model. In the model trained for 60 epochs, the maximum model weights for the IoU accuracy value evaluated in the validation images were recorded. Thus, model weights that provide the best training result were used. Afterward, the prediction performance was measured using the test dataset to evaluate the performance of the model on data that it had not seen before. The maximum rating metrics recorded for the Unet model are shown in Table 1.

As can be seen in the table, the model has very low scores. In Figure 7), the graph of the scores recorded during the training is given. As can be seen here, the model has difficulty in learning. Its performance on the test dataset is quite bad. For this problem, since the Unet model is insufficient, it was considered to use a deeper network. Therefore, it was considered to use the ResNet 152 structure instead of the standard convolutional neural network used in the encoder for feature extraction of Unet.

ResNet50 has a deep neural network architecture. It was considered to increase the performance of the Unet model when used as an encoder. Training was performed with previous model metrics and epoch count. In the model trained for 60 epochs, the maximum model weights for the IoU accuracy value evaluated in the validation images were recorded. Thus, model weights that provide the best training result were used. The maximum rating metrics recorded for the Unet-ResNet50 model are shown in (Table 2).

As can be seen in the table, there is a significant increase in educational performance. The performance of the model on the test dataset is seen to be quite successful. The success of the test dataset is parallel to the success of the training and validation dataset. Thus, it can be concluded that our model does not overlearn and has a good grasp of feature extraction. As can be seen in Figure 8, the model is quite successful in learning compared to the Unet model.

ResNet 152 has a deep neural network architecture. It has a deeper architecture than ResNet50. It was considered to increase the performance of the Unet model when used as an encoder. Training was performed with previous model metrics and epoch count. In the model trained for 60 epochs, the maximum model weights for the IoU accuracy value evaluated in the validation images were recorded. Thus, model weights that provide the best training result were used. The maximum rating metrics recorded for the Unet-ResNet152 model are shown in Table 3.

As can be seen in (Table 3, there is a significant increase in educational performance. The performance of the model on the test dataset is seen to be quite successful. The success of the test dataset is parallel to the success of the training and validation dataset. Thus, it can be concluded that our model does not overlearn and has a good grasp of feature extraction. As can be seen in Figure 9, the model is quite successful in learning compared to the Unet model.

After the success in model training, a visual evaluation of the model output of the test dataset was made. In Figure 10, you can see the original image, the masking it has, and the estimated masking output.

## 4. Discussion

In this work, image segmentation was performed using the Unet model. Model trainings were made for the Unet model by using different types of encoders for image segmentation, building extraction specifically. The accuracy evaluations, which are defined as intersection over union and dice loss metrics, of the performed model trainings on the test dataset are shown in Table 4.

As it can be seen in Table 4, ResNet architectures as a encoder for the Unet model outperform the standard CNN architectures. The ResNet architecture, which has a deeper architecture, has high accuracy in learning. Compared to ResNet50 and ResNet152, they have very close loss functions and close accuracy rates. The ResNet152 architecture has a deeper neural network than the ResNet50 architecture. The ResNet152 model contains more parameters due to its high layers. Therefore, it is at a disadvantage compared to the ResNet50 architecture in terms of speed and memory. The ResNet50 architecture offers a more suitable solution to the problem because it contains fewer parameters and higher accuracy than the ResNet152 architecture.

In Figure 11, a sample of our data can be seen from the Massachusetts building dataset with its true mask. At the right side, the output of the proposed and trained architecture is given, which was the best evaluated with respect to its test dataset by measuring intersection over union metric. As it can be seen there, the automatic building extraction is successfully performed on the test data. When the problems of the estimation are concerned, it can also be clearly seen that the detection of corners of the building is a quite hard work and estimated poorly. When only image segmentation is considered, the result is sufficient; however, for a building extraction, the result could be better, but there must be additional configuration so that the model can learn these buildings, which are mostly in a rectangular shape. It seems like this was the hardest part of image segmentation based on buildings.

## 5. Comparative Analysis

In 2016, Wang Shengsheng and his team used FCN-8s, SegNet, U-net, Deeplabv3, ENRU-Net models for building extraction in “Automatic Building Extraction from High-resolution Aerial Imagery via Fully Convolutional Encoder-Decoder Network With Non-local Block” [44]. The training results performed on the Massachusetts buildings dataset are shown in Table 5.

As seen in Table 5, the accuracy of the maximum intersection-over union function reached in the study is 73.02%. Compared with the Unet-ResNet50 model, the success of Unet-ResNet50 in building extraction is quite high. It can be said that the use of ResNet50 as an encoder shows a very high performance in extracting features.

In 2019, Pan Xuran and his team worked on FCN-8s, FCN-8s-SCA, and GAN-SCA models for building extraction from high-resolution antenna images [45]. In this study, the GAN-SCA model is proposed. The results obtained in the study performed on the Inria aerial image labeling dataset are shown in Table 6.

As can be seen in Table 6, the intersection-over union success of the GAN-SCA model presented by Pan Xuran and his team on the Inria aerial image labeling dataset is 74% on average. The performance of the Unet-ResNet50 model presented in this study is highly predictive in image segmentation. With the development of deep learning algorithms, building extraction studies on satellite images are also developing. There will be many developments and studies in this field in the future. The Unet-Resnet50 model proposed in this study seems quite satisfactory in today's conditions. Unet-ResNet50 offers the performance to perform building extraction from satellite images for a variety of practical applications such as land-use statistics and urban planning.

## 6. Conclusions

Unplanned urban settlements widely exist in less-developed countries. Automatic building extraction in the urban environment has long been challenging due to the high-density, complex surroundings, and various shapes of the buildings. In this work, deep learning algorithms, a sub-branch of artificial intelligence, were used to provide automatic building extraction in urban settlements. Thus, it is foreseen that planning can be made for urban structuring by extracting buildings in urban areas on satellite images. Image segmentation, one of the image processing methods, was preferred for building extraction. The widely used Unet model was used for image segmentation. Using the Massachusetts building dataset, the model was enabled to infer buildings on satellite images. The accuracy rates obtained in the trainings using different encoders of the Unet model were compared with the model performances. In the model evaluations, higher performance values were obtained with the ResNet architecture, which has a deeper architecture. As seen in Table 4, the Unet-ResNet50 model is much more effective in understanding the data than the Unet model. When the results are evaluated, the extraction of buildings over satellite images is provided very effectively with the ResNet50 model. City building mapping can be displayed quite clearly on the output images. In satellite images, there are hundreds of houses in a single image. When the margins of error in the corners of many buildings are evaluated over hundreds of houses, the 18% margin of error in the IoU function becomes significant. The margin of error here does not affect the location of the buildings. City building mapping can be clearly displayed as seen in the predicted building map shown in Figure 10.

## Figures and Tables

**Figure 1:** A sample from the dataset.

**Figure 2:** (a)Original image, (b) ground truth mask, and corresponding (c) one-hot encoded mask.

**Figure 3:** 256 × 256 cropped satellite image, mask, and one hot-encoded mask.

**Figure 4:** U-net architecture [1].

**Figure 5:** Training and test loss graph of 56- and 20-layer ResNet architecture on CIFAR 10. (a) The training error and (b) the test error [42].

**Figure 6:** Building block for residual learning [42].

**Figure 7:** Model train history of Unet.

**Figure 8:** Model train history of Unet-ResNet50.

**Figure 9:** Model train history of Unet-ResNet152.

**Figure 10:** Original satellite image, its true mask, and the estimated mask respectively.

**Figure 11:** Test result of ResNet152 architecture: original Image, its true mask, and the estimated mask.

**Table 1:** Maximum evaluate score for Unet model.

	Dice loss	IoU score	Accuracy	F1
Train data	0.153	0.531	0.780	0.7629
Valid data	0.611	0.663	0.871	0.860
Test data	0.932	0.212	0.719	0.603

**Table 2:** Maximum evaluate score for Unet-ResNet50 model.

	Dice loss	IoU score	Accuracy	F1
Train data	0.093	0.854	0.926	0.926
Valid data	0.090	0.860	0.926	0.925
Test data	0.108	0.822	0.902	0.900

**Table 3:** Maximum evaluate score for Unet-ResNet152 model.

	Dice loss	IoU score	Accuracy	F1
Train data	0.074	0.876	0.922	0.9225
Valid data	0.087	0.863	0.927	0.925
Test data	0.106	0.825	0.8996	0.897

**Table 4:** Model evaluation score on test dataset.

	Dice loss	IoU score	Accuracy	F1
Unet	3.3277	0.2316	0.719	0.603
Unet-ResNet50	0.108	0.822	0.902	0.900
Unet-ResNet152	0.106	0.825	0.8996	0.897

**Table 5:** Comparison with state-of-the-art models on Massachusetts building datasets [44].

Model	OA	IoU	F1
FCN	93.37	69.47	81.98
SegNet	93.84	72.1	93.78
U-net	93.63	69.97	82.14
Deeplab v3	93.01	68.55	81.34
ENRU-Net without APNB	94.12	72.77	84.24
ENRU-Net	94.18	73.02	84.41

**Table 6:** Experimental results on Inria aerial image labeling dataset [45].

Methods	Metrics	Austin	Chicago	Kitsap	Tyrol-w	Vienna	Overall
FCN-8s	IoU	67.98	67.98	53.17	68.13	72.03	98.05
	Acc.	95.47	95.47	99.01	97.52	92.38	95.16

FCN-8s-SCA	IoU	72.85	72.85	64.97	73.20	73.26	71.76
	Acc.	96.19	96.19	99.25	97.94	92.49	95.65

GAN-SCA	IoU	78.51	70.10	66.42	76.84	77.24	74.92
	Acc.	96.90	92.86	99.27	98.14	93.46	96.13

## Data Availability

The data used in this study can be extracted from https://www.kaggle.com/balraj98/massachusetts-buildings-dataset.

## References

[1] Wurm M., Stark T., Zhu X. X., Weigand M., Taubenböck H. (2019). Semantic segmentation of slums in satellite images using transfer learning on fully convolutional neural networks. *ISPRS Journal of Photogrammetry and Remote Sensing*.

[2] Bachofer F., Braun A., Adamietz F. (2019). Building stock and building typology of kigali, Rwanda. *Data*.

[3] Kuffer M., Persello C., Pfeffer K., Sliuzas R., Rao V. Do we underestimate the global slum population?.

[4] Kuffer M., Pfeffer K., Sliuzas R. (2016). Slums from space-15 Years of slum mapping using remote sensing. *Remote Sensing*.

[5] Li Y., Huang X., Liu H. (2017). Unsupervised deep feature learning for urban village detection from high-resolution remote sensing images. *Photogrammetric Engineering & Remote Sensing*.

[6] Olu-Ajayi R., Alaka H., Sulaimon I., Sunmola F., Ajayi S. (2022). Building energy consumption prediction for residential buildings using deep learning and other machine learning techniques. *Journal of Building Engineering*.

[7] Zhang G., Pan Y., Zhang L. (2022). Deep learning for detecting building façade elements from images considering prior knowledge. *Automation in Construction*.

[8] Wang Y., Li S., Teng F., Lin Y., Wang M., Cai H. (2022). Improved mask R-CNN for rural building roof type recognition from uav high-resolution images: a case study in hunan province, China. *Remote Sensing*.

[9] Yang H. (2022). Strategies for building robust prediction models using data unavailable at prediction time. *Journal of the American Medical Informatics Association*.

[10] Patino J. E., Duque J. C. (2013). A review of regional science applications of satellite remote sensing in urban settings. *Computers, Environment and Urban Systems*.

[11] Blaschke T. (2010). Object based image analysis for remote sensing. *ISPRS Journal of Photogrammetry and Remote Sensing*.

[12] Maggiori E., Tarabalka Y., Charpiat G., Alliez P. (2016). Convolutional neural networks for large-scale remote-sensing image classification. *IEEE Transactions on Geoscience and Remote Sensing*.

[13] Rodriguez-Galiano V. F., Chica-Olmo M., Abarca-Hernandez F., Atkinson P. M., Jeganathan C. (2012). Random Forest classification of Mediterranean land cover using multi-seasonal imagery and multi-seasonal texture. *Remote Sensing of Environment*.

[14] Huang B., Zhao B., Song Y. (2018). Urban land-use mapping using a deep convolutional neural network with high spatial resolution multispectral remote sensing imagery. *Remote Sensing of Environment*.

[15] Chen R., Li X., Li J. (2018). Object-based features for house detection from RGB high-resolution images. *Remote Sensing*.

[16] Carleer A. P., Debeir O., Wolff E. (2005). Assessment of very high spatial resolution satellite image segmentations. *Photogrammetric Engineering & Remote Sensing*.

[17] Duque J., Patino J., Betancourt A. (2017). Exploring the potential of machine learning for automatic slum identification from VHR imagery. *Remote Sensing*.

[18] Loures L., Vaz E. (2018). Exploring expert perception towards brownfield redevelopment benefits according to their typology. *Habitat International*.

[19] Zhu R., Wang Z., Ma Z., Wang G., Xue J.-H. (2018). LRID: a new metric of multi-class imbalance degree based on likelihood-ratio test. *Pattern Recognition Letters*.

[20] Li X., Ma Z., Peng P. (2018). Supervised latent Dirichlet allocation with a mixture of sparse softmax. *Neurocomputing*.

[21] Zhu F., Ma Z., Li X. (2019). Image-text dual neural network with decision strategy for small-sample image classification. *Neurocomputing*.

[22] Hodgson M. E. (1988). Reducing the computational requirements of the minimum-distance classifier. *Remote Sensing of Environment*.

[23] Huang K.-Y. (2002). The use of a newly developed algorithm of divisive hierarchical clustering for remote sensing image analysis. *International Journal of Remote Sensing*.

[24] Pal M. (2005). Random forest classifier for remote sensing classification. *International Journal of Remote Sensing*.

[25] Li Y., Qi H., Dai J., Ji X., Wei Y. Fully convolutional instance-aware semantic segmentation.

[26] Lo S.-C. B., Chan H.-P., Lin J.-S., Li H., Freedman M. T., Mun S. K. (1995). Artificial convolution neural network for medical image pattern recognition. *Neural Networks*.

[27] Zand R. (2017). R-DBN: A resistive deep belief network architecture leveraging the intrinsic behavior of probabilistic devices. https://arxiv.org/abs/1710.10903.

[28] Miao Y., Gowayyed M., Metze F. EESEN: end-to-end speech recognition using deep RNN models and WFST-based decoding.

[29] Yu Y., Liu F. (2018). Aerial scene classification via multilevel fusion based on deep convolutional neural networks. *IEEE Geoscience and Remote Sensing Letters*.

[30] Canetti A., Garrastazu M. C., Mattos P. P. d., Braz E. M., Pellico Netto S. (2018). Understanding multi-temporal urban forest cover using high resolution images. *Urban Forestry and Urban Greening*.

[31] Milan A. (2018). An integrated framework for road detection in dense urban area from high-resolution satellite imagery and Lidar data. *Journal of Geographic Information System*.

[32] Wang Y., Chen A. S., Fu G., Djordjević S., Zhang C., Savić D. A. (2018). An integrated framework for high-resolution urban flood modelling considering multiple information sources and urban features. *Environmental Modelling & Software*.

[33] Tane Z., Roberts D., Koltunov A., Sweeney S., Ramirez C. (2018). A framework for detecting conifer mortality across an ecoregion using high spatial resolution spaceborne imaging spectroscopy. *Remote Sensing of Environment*.

[34] Li Y., Ye D. (2018). Greedy annotation of remote sensing image scenes based on automatic aggregation via hierarchical similarity diffusion. *IEEE Access*.

[35] Basu S., Ganguly S., Mukhopadhyay S., DiBiano R., Karki M., Nemani R. Deepsat: a learning framework for satellite imagery.

[36] Van Etten A., Lindenbaum D., Bacastow T. M. (2018). Spacenet: a remote sensing dataset and challenge series. https://arxiv.org/abs/1807.01232.

[37] Yang Y., Newsam S. Bag-of-visual-words and spatial extensions for land-use classification.

[38] Cheng G., Yang C., Yao X., Guo L., Han J. (2018). When deep learning meets metric learning: remote sensing image scene classification via learning discriminative CNNs. *IEEE Transactions on Geoscience and Remote Sensing*.

[39] Zhang C., Sargent I., Pan X. (2018). An object-based convolutional neural network (OCNN) for urban land use classification. *Remote Sensing of Environment*.

[40] Kaggle Web Page (2021). Massachusetts buildings dataset. https://www.kaggle.com/balraj98/massachusetts-buildings-dataset,02/12/2021.

[41] Ronneberger O., Fischer P., Brox T. (2015). U-net: convolutional networks for biomedical image segmentation. https://arxiv.org/abs/1505.04597.

[42] He K., Zhang X., Ren S., Sun J. Deep residual learning for image recognition.

[43] Wikipedia Web Page (2021). Sorensen-dice coefficient. https://en.wikipedia.org/wiki/Sørensen–Dice_coefficient,02/12/2021.

[44] Wang S., Hou X., Zhao X. (2020). Automatic building extraction from high-resolution aerial imagery via fully convolutional encoder-decoder network with non-local block. *IEEE Access*.

[45] Pan X., Yang F., Gao L. (2019). Building extraction from high-resolution aerial imagery using a generative adversarial network with spatial and channel attention mechanisms. *Remote Sensing*.

